The article "Research on Classification of COVID-19 Chest X-Ray Image Modal Feature Fusion Based on Deep Learning" was published in 2021. Journal: J Healthc Eng.

# Research on Classification of COVID-19 Chest X-Ray Image Modal Feature Fusion Based on Deep Learning

**DOI:** 10.1155/2021/6799202

**Published:** 2021-08-24

**Authors:** Dongsheng Ji, Zhujun Zhang, Yanzhong Zhao, Qianchuan Zhao

**Affiliations:** ^1^School of Computer and Communication, Lanzhou University of Technology, Lanzhou 730000, China; ^2^Center for Intelligent and Networked Systems (CFINS), Department of Automation, Tsinghua University, Beijing 100084, China

## Abstract

Most detection methods of coronavirus disease 2019 (COVID-19) use classic image classification models, which have problems of low recognition accuracy and inaccurate capture of modal features when detecting chest X-rays of COVID-19. This study proposes a COVID-19 detection method based on image modal feature fusion. This method first performs small-sample enhancement processing on chest X-rays, such as rotation, translation, and random transformation. Five classic pretraining models are used when extracting modal features. A global average pooling layer reduces training parameters and prevents overfitting. The model is trained and fine-tuned, the machine learning evaluation standard is used to evaluate the model, and the receiver operating characteristic (ROC) curve is drawn. Experiments show that compared with the classic model, the classification method in this study can more effectively detect COVID-19 image modal information, and it achieves the expected effect of accurately detecting cases.

## 1. Introduction

In December 2019, the first case of the novel coronavirus pneumonia (COVID-19) was confirmed in Wuhan, China. In just two months, the number of confirmed cases rose to nearly 1000, with more than 5000 suspected cases. By September 2020, the novel coronavirus pneumonia epidemic had spread across the world, and the number of confirmed cases increased daily.

In the early stages of the epidemic, people knew very little about the novel coronavirus. According to the “Novel Coronavirus Diagnosis and Treatment Plan for Pneumonia infected by Bat disease (Trial Version 5),” released by the China National Health Commission on February 4, 2020, and the explanation by Dr. Nanshan Zhong of the COVID-19 epidemic, the novel coronavirus and SARS bat-like coronavirus (Bat-SL-CoVZC45) have over 85% homologies, belonging to the same family but not being the same kind [1]. On February 9, 2020, the team of academician Zhong Nanshan published a paper on the analysis of the clinical characteristics of the novel coronavirus pneumonia in China [2]. The study of 1099 positive patients and analysis of clinical samples revealed a number of clinical features of the novel coronavirus pneumonia infection, emphasizing the main symptoms and radiological characteristics of the patient. In the diagnosis and treatment plan of the “Novel Coronavirus Infection Pneumonia Diagnosis and Treatment Plan (Trial Version 7),” issued by the National Health Commission [3], in addition to an incubation period of 1–14 days of isolation, observation based on epidemiological investigations, according to the clinical manifestations of pneumonia symptoms, characteristics of disease signs, laboratory nasopharyngeal swabs, nucleic acid test results of negative/positive, and effective oxygen therapy combined with antiviral and antimicrobial therapy, the most important diagnostic criterion is chest imaging.

The article "Research on Classification of COVID-19 Chest X-Ray Image Modal Feature Fusion Based on Deep Learning" was published in 2021. Journal: J Healthc Eng.

For the initial research on COVID-19, Shan et al. proposed an automatic segmentation and quantification system based on deep learning, using image segmentation theory to study the chest computer tomography (CT) infection area and the overall structure of the lungs, and man-machine loop optimization to annotate each case [4]. Wang et al. from the Cancer Hospital of Tianjin Medical University used deep learning to extract COVID-19 image features, established a learning model to analyse positive cases and provided a theoretical basis for the timely and accurate diagnosis of COVID-19 [5]. Experts from the Affiliated Hospital of Huazhong University of Science and Technology used three-dimensional CT to detect the novel coronavirus pneumonia and a three-dimensional neural network based on weakly supervised deep learning to classify positive and negative cases to quickly identify COVID-19 cases [6]. Researchers such as Asmaa and Mohammed from Arthurs University and Birmingham City University, aiming at the high availability of COVID-19 annotated image datasets, used convolutional neural networks (CNNs) to identify and classify novel coronavirus pneumonia images and a class decomposition mechanism to study its class boundary to deal with irregularities in the dataset, with good results [7]. Li used deep CNNs to study positive cases of chest CT image data of patients with novel coronavirus pneumonia [8]. Rehman et al. used pretrained knowledge and transfer learning to distinguish COVID-19 disease from viral pneumonia, bacterial pneumonia, and healthy people, so as to develop an effective diagnostic method [9].

With the development of the epidemic, machine learning technology and deep learning technology have been applied in the detection of COVID-19 patients. Wang et al. applied an Inception network to CT to detect COVID-19 [5]. Asif et al. used a transfer learning inception V3 model to detect COVID-19 chest X-ray images, proving that the transfer learning method is robust and easy to expand for COVID-19 detection [10]. Song et al. used an improved version of the ResNet50 pretrained network to accurately classify healthy people, COVID-19, and bacterial pneumonia [11]. Loey et al. used the GooLeNet pretraining model to classify COVID-19, bacterial pneumonia, viral pneumonia, and normal people, with an 80.6% accuracy rate [12]. Rahimzadeh and Attar used Xception and ResNet50V2 to develop a tandem CNN to classify chest X-ray images of COVID-19 with a correct rate of 99.56% [13]. Hassanien et al. combined a multilevel threshold with a support vector machine (SVM) system to classify X-ray images of COVID-19-infected persons with high accuracy [14]. Alqudah et al. used machine learning techniques such as SVM, CNN, and random forest (RF) to classify COVID-19 X-ray images, with high accuracy [15]. Osi proved that RF predicts COVID-19 results better than linear discriminant analysis (LDA) and SVM [16]. Kumar et al. proposed a classification model based on deep transfer learning, integrating DenseNet121 and SquezeNet 1.0 (DeQueezeNet) to extract the importance of various impact features from COVID-19 X-ray images and effectively classify COVID-19 cases [17]. Abbas et al. verified and adjusted a deep CNN called decomposition, transmission, and synthesis (DeTrac) to classify COVID-19 chest X-ray images. DeTraC is a class decomposition mechanism for studying image datasets, whose boundary can handle any irregularities [7]. Apostolopoulos et al. used five CNN variants to multiclassify COVID-19 images with 93.48% accuracy [18]. Horry et al. used VGG16 and VGG19 models to detect COVID-19, with recall and precision rates both equal to 80% [19]. Sethy and Behera introduced a deep learning method that uses chest X-ray images to classify patients infected with COVID-19 [20]. The program uses nine pretrained models for feature extraction and SVMs for classification. The prediction accuracy of ResNet50-plus SVM was better than that of other models, with F1-scores of 95.38% and 95.52%, respectively.

The article "Research on Classification of COVID-19 Chest X-Ray Image Modal Feature Fusion Based on Deep Learning" was published in 2021. Journal: J Healthc Eng.

## 2. Materials and Methods

The detection of COVID-19 in this article requires several stages, as shown in Figure 1. The original X-ray image is preprocessed, including size adjustment, rotation, position translation, cross-cutting transformation, scaling, and flip processing. The dataset is then divided into training and validation (test) sets. The preprocessed data are used to extract the modal feature information of the X-ray images through pretraining models by transfer learning, and this is input to the fully connected (FC) layer and trained after fusion. The first two layers of the FC layer contain 512 hidden units, followed by the ReLU activation function, and the last layer contains a hidden unit, followed by the sigmoid activation function, which is used to detect COVID-19. The performance of the system is evaluated by indices such as accuracy, recall rate, precision, and F1-score.

### 2.1. Dataset

Chest imaging is commonly used in medicine, and it plays an important role in the detection of COVID-19. Through the diagnosis of chest imaging, medical staff can more accurately grasp the imaging modal characteristics of COVID-19 cases, such as multiple small patchy shadows and interstitial changes in the early stage, which are obvious outside the lungs. It then develops into multiple ground glass and infiltration shadows in both lungs. In severe cases, lung consolidation and pleural effusion are rare. It has important guiding value for accurately judging the condition and its development, formulating treatment plans, and evaluating prognoses. There are many COVID-19 datasets, but the number of samples is small. The experiment collected 4099 COVID-19 chest X-rays on Kaggle, consisting of 3278 in a training set and 821 in a validation (test) set.  Figure 2 shows several chest X-ray images in the dataset, where (a) is from a COVID-19 patient and (b) is from a healthy person.

Table 1 shows that the training set of the COVID-19 dataset is 3278 X-ray images, and the test set only has 821 X-ray images. The data distribution is relatively unbalanced. If the training validation set is divided by a ratio of 0.3, serious overfitting will occur. Therefore, a division ratio of 0.2 is most appropriate. In the experiment, the label of a normal person is set to 0 and the label of a COVID-19 patient is 1. Table 1 shows the distribution of the COVID-19 dataset.

### 2.2. Transfer Learning

Transfer learning improves learning by transferring knowledge from related tasks that have been learned, i.e., transferring learned and trained parameters to a new model to help with its training [21]. The architecture of deep learning models is complex and data dependent, requiring much data to train them. Much COVID-19 data are published online, but the number of samples is small, making it difficult to train a deep learning model from start to finish. Transfer learning can facilitate the training of such a small sample dataset to achieve the research purpose.

Apostolopoulos et al. adopted transfer learning to detect the performance of different models in a small sample of pneumonia image datasets [18]. Rafi [22] used chest X-ray images to identify patients with COVID-19, using transfer learning methods to train DenseNet121 and ResNet152 series models. Taresh et al. discussed the effectiveness of artificial intelligence in the rapid and reliable detection of COVID-19 based on chest X-ray images and applied transfer learning technology to detect COVID-19 from chest radiographs [23]. Majeed et al. compared 12 transfer learning CNNs in the detection of COVID-19 from chest X-rays [24].

The article "Research on Classification of COVID-19 Chest X-Ray Image Modal Feature Fusion Based on Deep Learning" was published in 2021. Journal: J Healthc Eng.

The COVID-19 samples collected for our experiment were limited. To obtain better experimental results, different CNN models trained on ImageNet, a database of approximately 14 million images, were used to train the COVID-19 dataset.

### 2.3. Convolutional Neural Network Model

Xception [25] is an improvement of Inception V3, replacing its convolution operation with depthwise separable convolution, which divides traditional convolution into the steps of depthwise and pointwise convolution.

The InceptionResNetV2 [26] model is a CNN with top accuracy on the ILSVRC image classification benchmark. It is based on Google's Inception V3 model and draws on the ideas of ResNet [27], a 152-layer neural network successfully trained by using the ResNet Unit. The error rate on Top5 is 3.57%. It has fewer parameters than VGGNet, and the effect is outstanding. It introduces the idea of residual learning, which effectively solves the problem of network degradation.

The VGG [28] family is used in face recognition and image classification, where VGG19 has better performance. VGG19 has 19 hidden layers, consisting of 16 convolutional layers and three fully connected layers. The input is set to 224 × 224 RGB images. The RGB average of all images is calculated on the training set image, and the image is passed as input and enters the VGG19 convolutional network.

DenseNet [29] builds a connection relationship between layers, makes full use of features, and further alleviates the problem of gradient disappearance. The use of a bottleneck layer, translation layer, and smaller growth rate makes the network narrower, reduces the parameters, effectively suppresses overfitting, and reduces calculation.

### 2.4. Fusion Model

The experimental architecture uses pretrained Xception, ResNet152, DenseNet201, VGG19, and InceptionResNetV2 CNN to extract the feature information of COVID-19 X-ray lung images. Each network has three FC layers, where the last layer is FC for classification. In this experiment, the FC layer behind each network is replaced by the global average pooling layer, which can effectively reduce the training parameters. The dataset contains chest X-ray images of COVID-19 cases and healthy people. We set the label of COVID-19 images to 1 and images of healthy people to 0, for training and evaluating the model.

The experiment uses these five CNN structures to extract feature maps. As shown in Figure 3, each model is followed by a global average pooling layer and a flatten layer. The input feature maps are “flattened”; i.e., the multidimensional input is one dimensional, and the output is a one-dimensional feature vector that is passed through dropout, which is used to avoid overfitting in training. The dropout is set to 0.5 and finally input into the designed FC layer. The FC layer has three layers. The first two are dense layers with 512 hidden units, and the last is a dense layer with one hidden unit. The purpose is to detect COVID-19 patients.

The article "Research on Classification of COVID-19 Chest X-Ray Image Modal Feature Fusion Based on Deep Learning" was published in 2021. Journal: J Healthc Eng.

### 2.5. Evaluation Standard

The following indicators are used to measure the performance of the cascade model system. TP is a correctly predicted COVID-19 case, FP is misclassified as a COVID-19 case, TN is a normal person that is correctly classified, and FN is misclassified as a normal person. The performance of the proposed cascade model system is measured by accuracy, precision, recall and F1-score. The mathematical expression of the evaluation index parameters is as follows:

(1) $$\begin{array}{c} \text{Accuracy}=\frac{\text{TP}+\text{TN}}{\text{TN}+\text{FP}+\text{TP}+\text{FN}},\\ \text{Precision}=\frac{\text{TP}}{\text{FP}+\text{TP}},\\ \text{Recall}=\frac{\text{TP}}{\text{FN}+\text{TP}},\\ \text{F}1‐\text{score}=\frac{2*\text{precision}*\text{recall}}{\text{precision}+\text{recall}}. \end{array}$$

## 3. Results and Discussion

All experiments are carried out on the kaggle server, using the Tesla P100-PCIE-16 GB GPU graphics card and python language tensorFlow/keras framework.

### 3.1. Data Preprocessing and Training of Parameter Settings

We discuss and analyse the experimental results. Before training the model, we normalized the training and validation (test) datasets to decimal values between (0, 1) or (1, 1), so as to make training more convenient and faster. Since the experiment used small samples, the training and validation datasets were scaled. The input size of the VGG19, DenseNet201, and ResNet152 network models was 224 × 224, so the input image size was set to that size. Similarly, the input size of Xception and InceptionResNetV2 was set to 299 × 299. In the experiment, all images were rotated, zoomed, cut, and reversed in an anticlockwise direction to facilitate training. The parameter settings for preprocessing and training are shown in Table 2.

In the preprocessing stage, all parameters were set the same to enhance the sample data. In the training phase, we first set empirical values for some main parameters, e.g., a learning rate of 0.01 and batch size of 128, with 10 epochs and 128 nodes in the first two layers of the FC layer. In the training process, loss converges according to the learning rate. Loss that does not converge is probably due to too high learning rate, and slow convergence usually means the learning rate is set too low. In this experiment, the learning ability of the model was best with a learning rate of 0.001. When the accuracy is very low, the batch size can be reduced while keeping the number of epochs unchanged, which will improve the accuracy because the larger the batch size, the faster the processing. In the case of constant epochs, the batch size needs to be reduced to achieve the same accuracy. After many adjustments and experiments, the batch size and number of epochs were set to 16 and 500, respectively (except for model 2, with 1000 epochs). Underfitting or overfitting may occur during training, and the number of nodes in the FC layer and the dropout size can be adjusted appropriately. The number of nodes in the FC layer and the dropout was set to 512 and 0.5, respectively, but the loss curves of training and testing showed severe jitter, so momentum was added to reduce jitter, and this was set to 0.9 for better model learning.

The article "Research on Classification of COVID-19 Chest X-Ray Image Modal Feature Fusion Based on Deep Learning" was published in 2021. Journal: J Healthc Eng.

The stochastic gradient descent (SGD) optimizer minimizes or maximizes the loss function by training and optimizing model parameters, and the neural network selects samples randomly instead of rigidly for gradient calculation when performing gradient descent. SGD performs parameter updates for each training sample *x*^(*i*)^ and label *y*^(*i*)^:

(2) $$\begin{array}{c} \theta =\theta -\eta *\nabla_{\theta }J\left(\theta ;x^{\left(i\right)};y^{\left(i\right)}\right),\;i=1,2,3,\ldots ,Ν. \end{array}$$

The learning rate *η* determines the size of the steps taken to reach the (local) minimum, where *J*(*θ*) is the objective function, *θ* is the model parameter, and ∇*J*(*θ*; *x*^(*i*)^; *y*^(*i*)^) is the gradient. The objective function *J*(*θ*) takes parameter *θ* of the model by updating the parameters in the opposite direction of the gradient of the objective function.

The experimental loss function is binary cross entropy, which is generally used for binary classification, and describes the difference between the predicted and true values of the model. The larger the value, the less the similarity. The binary cross-entropy loss function formula is as follows:

(3) $$\begin{array}{c} H_{p}\left(q\right)=-\frac{1}{N}\sum_{i=1}^{N}y_{i}\log\left(p\left(y_{i}\right)\right)+\left(1-y_{i}\right)*\;\log\left(1-p\left(y_{i}\right)\right),\;i=1,2,3,\ldots ,N, \end{array}$$

where *N* is the number of categories, *y* is the label (1 for COVID-19 and 0 for healthy persons), and *p*(*y*) is the predicted probability of COVID-19 in all *N* samples. For each COVID-19 case (*y* = 1), it adds log(*p*(*y*)) to the loss, which means it is the logarithmic probability of COVID-19. It adds log (1 − *p* (*y*)) for each healthy person (*y* = 0), so it is the log probability of a healthy person.

The article "Research on Classification of COVID-19 Chest X-Ray Image Modal Feature Fusion Based on Deep Learning" was published in 2021. Journal: J Healthc Eng.

### 3.2. Summary of Pretrained Convolutional Neural Network Architectures Used in This Study

Table 3 shows the CNN architecture information for this study. It can be seen that ResNet50 has the smallest number of layers, at 50, and model 2, which contains 5 CNN architectures, has the most. The size of Xception is 88 MB, which is the smallest of these CNN structures, and model 2 is the largest. ResNet50 has 23.52 M parameters, which is the smallest. Model 2 has the largest number of parameters. Table 3 gives the details of the pretraining architecture used in this study.

## 4. Results and Discussion

This article uses ResNet50, ResNet152, Xception, InceptionResNetV2, and cascade models 1 and 2 to distinguish between COVID-19 and healthy people. These models were trained and tested under the same conditions (dataset, FC layer, and parameter settings). The performance of the network models was compared according to the accuracy, precision, recall, and F1-score of the test set, which, according to Table 3, were 96%, 96.1%, 96.42%, and 95.5%, respectively, for model 2. These were higher for other single models and model 1 because a single deep learning network will lose some detailed feature information when extracting COVID-19 lung modal feature information, eventually leading to poor classification results. However, model 2 uses several single models to extract the modal features of the COVID-19 lung image in parallel, which can effectively retain the detailed feature information of the image, for a better final classification effect than a single model.

To better understand the model training process, the experiment extracted the feature maps output from the first layer and some convolutional layers of Xception, ResNet152, DenseNet201, VGG19, and InceptionResNetV2. According to the feature map output from the first layer of each CNN model, we compared the chest X-rays of COVID-19 patients and healthy people. We found that the area of interest of the CNN model was the yellow area, and the model has more areas of interest on COVID-19 chest X-rays than for healthy people.  Figure 4 shows some of the extracted feature maps. The VGG19 first layer output area of interest is mainly white, the chest X-ray of COVID-19 is slightly whiter, and the chest X-ray of healthy people is basically not white.

First, the experiment uses ResNet50 to detect COVID-19. The loss and accuracy curves of the model are shown in Figure 5(a). The experimental training accuracy reaches 91.70%, and the validation accuracy reaches 93.17%. It can be seen from the figure that the training and validation accuracy curves basically overlap, but they can only reach about 91.70%, and the training loss has become flat, about 0.23. The experiment uses RenNet152 to detect COVID-19 patients. The training accuracy of the model is 92.83%, and the validation accuracy is 93.39%. The loss and accuracy curves of the model are shown in Figure 5(b). In analysis (b), the training and validation accuracy of ResNet152 are higher than those of ResNet50, and the loss curve effect is also better. Using Xeption to detect COVID-19 patients, the model has a training accuracy of 93.63% and a validation accuracy of 94.39%. The loss and accuracy curves of the model are shown in Figure 5(c). The loss and Accuracy graphs of the Xception model are better than ResNet50 and ResNet152. It can be said that its training effect is very good and the loss has been flat. Using InceptionResnetV2 to detect COVID-19 patients, the model has a training accuracy of 89.27% and a validation accuracy of 90.22%. The loss and accuracy curves of the model are shown in Figure 5(d). The experiment uses Xception, ResNet152, DenseNet201, VGG19, and InceptionResNetV2 model feature fusion, the training accuracy reaches 96.58%, and the validation accuracy is 96.00%.  Figure 5(f) is the loss and accuracy curves of the model architecture.  Figure 5(e) uses the Xception, ResNet50, and Inception V3 cascade mode to detect COVID-19, training accuracy rate is 95.49%, and validation accuracy rate is 94.76%, slightly lower than those of the cascade model using five models.

The article "Research on Classification of COVID-19 Chest X-Ray Image Modal Feature Fusion Based on Deep Learning" was published in 2021. Journal: J Healthc Eng.

Table 4 is the evaluation index results of the experimental validation (test) set. It can be seen that the accuracy, precision, recall, and F1-score of ResNet50 on the test set are 93.17%, 95%, 94.43%, and 93.83%, respectively. Compared with ResNet50, the accuracy, precision, recall, and F1-score of model 2 have increased by 2.83%, 1.1%, 1.99%, and 1.67%, respectively. The accuracy, precision, recall, and F1-score of ResNet152 on the test set are 93.39%, 95.87%, 94.84%, and 95.11%, respectively. Compared with ResNet152, model 2's accuracy, precision, recall, and F1-score increased by 2.61%, 0.23%, 1.58%, and 0.39%, respectively. The accuracy, precision, recall, and F1-score of Xception on the test set are 94.39%, 95.79%, 93.86%, and 94.46%, respectively. Compared with Xception's accuracy, precision, recall, and F1-score, those of model 2 increased by 1.61%, 0.31%, 2.56%, and 1.04%, respectively. The accuracy, precision, recall, and F1-score of InceptionResNetV2 on the test set are 90.22%, 95.06%, 91.02%, and 92.22%, respectively. Compared with InceptionResNetV2's accuracy, precision, recall, and F1-score, those of model 2 increased by 5.78%, 1.04%, 5.4%, and 3.73%, respectively. The accuracy, precision, recall, and F1-score of model 1 on the test set are 94.76%, 95.45%, 96.02%, and 94.99%, respectively. Compared with model 1's accuracy, precision, recall, and F1-score, those of model 2 increased by 1.24%, 0.65%, 0.4%, and 0.5%, respectively. It can be noticed that all the indicators of model 2 have been improved.

The article "Research on Classification of COVID-19 Chest X-Ray Image Modal Feature Fusion Based on Deep Learning" was published in 2021. Journal: J Healthc Eng.

The receiver operating characteristic (ROC) curve is an evaluation index for binary classification problems, and the area under the curve (AUC) is a measure of the ability of the classifier to classify. The higher the AUC, the better the model's performance in distinguishing between positive and negative classes.  Figure 6 shows the ROC curves of six CNN architectures. The classifier uses a fully connected layer and an RF. It can be found that the classification effect of the FC layer is better than the classification effect of the random forest. When using fully connected layer classification, the AUC of InceptionResNetV2 is 0.966, the lowest among these models. The highest is model 1 with an AUC of 0.989. Model 2 AUC is 0.987, Xception AUC is 0.984, ResNet152 AUC is 0.981, and ResNet50 AUC is 0.977, among which model 2 is 0.002 lower than model 1, but the classification effect is similar.

The results of the six CNN architectures on the test dataset show that model 2 has higher accuracy, precision, recall, and F1-scores than the other algorithms, and the AUC value differs by only 0.002 from model 1. From these data, it is concluded that model 2 has a good classification effect on COVID-19 and healthy people. Compared with other models, model 2 has better adaptability to the modal characteristics of COVID-19 lungs and can improve the accuracy on the test set. This is because the ResNet50, ResNet152, Xception, and InceptionResNetV2 models lose some detailed information when extracting features, and this varies by model according to the network structure. Models 1 and 2 have a cascade architecture, which can integrate the feature information extracted by a single model, and the final classification result is good. Model 1 is composed of the ResNet50, Xception, and Inception v3 models, and model 2 is composed of the Xception, ResNet152, DenseNet201, VGG19, and InceptionResNetV2 models. So, model 2 can save more feature information, and the final classification result is better. As can be seen in Table 3, although the ResNet50 network has only 50 layers, there are only 23.52 M parameters, so the characteristics of COVID-19 are prone to be lost, and the test accuracy is not high. The Xception network has 126 layers and only 22.91 M parameters. It can extract deeper features, but it loses much COVID-19 feature information. The ResNet152 network has 152 layers and 60.42 M parameters, and the detection effect is not ideal because the residual network can be no deeper, which will cause convergence to fail on the COVID-19 dataset. The InceptionResNetV2 network has 55.87 M parameters, but the number of network layers reaches 572, so a large dataset is required to train the network, and the amount of data in this experiment is small, causing poor results. Model 2 combines the advantages of the VGG19, DesenNet201, Xception, ResNet152, and InceptionResNetV2 networks, so the better the fitting ability on the COVID-19 dataset, the better the classification effect.

The article "Research on Classification of COVID-19 Chest X-Ray Image Modal Feature Fusion Based on Deep Learning" was published in 2021. Journal: J Healthc Eng.

Table 5 shows the calculation time required for training and testing of all models. It can be seen that model 2 takes 1503.67 s and 138.66 s, respectively, for training and testing, more than the other models. The more complex the network structure, the longer it takes to extract features, so model 2 takes more time, and it has a higher accuracy rate. It can be noticed that ResNet50 takes the least training time, 418.91 s, and the test time of InceptionResNetV2 is the least, at 52.44 s, but their accuracy is very low.

We compare our research with recent work, with results in Table 6. Sethy and Behera used ResNet50, with SVM instead of deep learning classifiers for classification, and its accuracy and F1-score were 95.33% and 95.34%, respectively [20]. Ismael and Şengür used 6 pretrained CNN models to extract the depth features of 180 COVID-19 and 200 healthy X-ray images and classified them with SVM. ResNet50+SVM achieved an accuracy of 94.7%, highest of all their results [30]. Sethy and Ismael used the same method to classify COVID-19 and healthy people, and the accuracy obtained is very similar to F1-score, but the accuracy is lower than that of model 2, and the recall of the method proposed by Ismael (91%) is lower than that of model 2 (96.42%). Hemdan et al. used seven deep CNN models with different structures to classify COVID-19 and healthy people [31]. VGG19 and DenseNet201 showed similarly good classification performance, and accuracy, F1-score, precision, and recall were 90%, 91.5%, and 90%, respectively, which were far lower than those of model 2 because the experiment only used 50 COVID-19 images to verify the performance of the model. Sahinbas and Catak proposed that the pretrained VGG16 model has a poor classification effect [32]. The accuracy, F1-score, precision, and recall are all 80%, which are much lower than the indicators of model 2. Das used the cascade network of DenseNet201, ResNet50V2, and Inception v3 to classify COVID-19 and healthy people, with only 91.62% accuracy [33]. Kumar et al. proposed a model structure based on the fusion of DenseNet121 and SquezeNet1.0, called DeQueezeNet [17]. The precision and accuracy of the model were 94.52% and 90.48%, respectively. Jaiswal et al. proposed a transfer learning approach on a pruned EfficientNet-based model for the detection of COVID-19 cases [34]. The accuracy of the binary classification of this method on the X-ray dataset reached 96%, which is consistent with the accuracy of model 2, but the F1-score, precision, and recall indicators were all lower.

The article "Research on Classification of COVID-19 Chest X-Ray Image Modal Feature Fusion Based on Deep Learning" was published in 2021. Journal: J Healthc Eng.

According to the analysis and discussion of the evaluation criteria of the comparative research algorithm on the test set in this article, the accuracy, precision, recall, and F1-score of model 2 are higher than those of comparative research algorithms, showing that model 2 can more effectively distinguish COVID-19 patients from healthy people and is considered to be a major in-depth architecture. This article also compares and discusses with recent research results; in the analysis of recent work in Table 6, it can be observed that the performance of all indicators of model 2 is better than that of other research methods. Only the COVIDPEN network of Jaiswal has a classification accuracy of 96%, which is the same as that of model 2. Therefore, in the end, compared with other studies, model 2 showed good performance. From these aspects, model 2 is seen to show good performance in distinguishing between COVID-19 patients from healthy people.

## 5. Conclusions

CT and X-rays are effective tools for diagnosing and evaluating COVID-19. We used four CNN models and two cascaded network models to divide X-ray samples into two categories: COVID-19 and healthy people. We applied these model architectures for feature extraction and classified categories through an FC layer. Experimental results showed that, under the same conditions, cascade network model 2 was best for classifying COVID-19 and healthy people. It could significantly improve classification performance, with accuracy of 96%, F1-score of 95.5%, 96.10% precision, 96.42% recall, and 98.7% AUC. We discussed and compared our research and recent work. The results showed that model 2 is better than other models in classifying COVID-19 and healthy people, can accurately classify them, and can assist doctors in the rapid detection of COVID-19. We concluded from these two aspects that model 2 is well distinguished between COVID-19 patients and healthy people and could help reduce the workload of doctors in detecting COVID-19 cases.

The article "Research on Classification of COVID-19 Chest X-Ray Image Modal Feature Fusion Based on Deep Learning" was published in 2021. Journal: J Healthc Eng.

The method proposed in this paper can be applied to the classification of modal characteristics of other lung diseases. Patients with pulmonary edema and lung tumours have pulmonary modal characteristics such as ground glass shadow and infiltration shadow. Early lung disease usually has infiltration shadow, and then, ground glass shadow appears. These phenomena can determine the severity of lung disease. The algorithm in this study is more sensitive to the modal characteristics of the new coronavirus pneumonia, which has similar modal characteristics to pulmonary edema and lung tumours, so the algorithm can be applied to the classification of modal characteristics of lung diseases. The algorithm can also be extended to classify magnetic resonance imaging (MRI), which is of great value in the differential diagnosis of liver cancer, and can clearly show the characteristics of tumour foci. Although the algorithm in this paper cannot identify tumour features, it is sensitive to obvious modal features and can be applied to MRI image classification of liver cancer through small-sample training in the later stage.

The proposed method has major limitations. The experiment only applies to X-ray images, and not CT images, because X-ray images are RGB and CT images are grayscale. This experiment can only be used to classify COVID-19 patients and healthy people, and it cannot classify COVID-19 and general pneumonia. We will next focus on the classification of COVID-19, bacterial pneumonia, and viral pneumonia.

## Figures and Tables

**Figure 1:** The overall architecture of the COVID-19 classification framework.

**Figure 2:** Partial sample of the COVID-19 dataset. (a) A chest X-ray of COVID-19. (b) A chest X-ray of healthy people.

**Figure 3:** Cascade network model diagram.

**Figure 4:** Feature map output by the convolutional layer.

**Figure 5:** Accuracy and loss curves of five convolutional neural network structures. (a) ResNet50, (b) ResNet152, (c) Xception, (d) InceptionResNetV2, (e) ResNet50, Xception, and InceptionV3 cascade structure, and (f) Xception, ResNet152, DenseNet201, VGG19, and InceptionResNetV2 cascade structure.

**Figure 6:** Receiver operating characteristic curves of six convolutional neural network structures. (a) ResNet50. (b) ResNet152. (c) Xception. (d) InceptionResNetV2. (e) ResNet50, Xception, and InceptionV3. (f) Xception, ResNet152, DenseNet201, VGG19, and InceptionResNetV2.

**Table 1:** Distribution of the COVID-19 dataset.

Category	Training set	Validation (test) set	Total
Normal	889	223	1112
COVID-19	2389	598	2987
Total	3278	821	4099

**Table 2:** Preprocessing and training phase parameters.

Parameters	Model					
	ResNet50	ResNet152	Xception	Inception ResNetV2	Model 1	Model 2
Learning rate	1*e* − 3	1*e* − 3	1*e* − 3	1*e* − 3	1*e* − 3	1*e* − 3
Batch	16	16	16	16	16	16
Optimizer	SGD	SGD	SGD	SGD	SGD	SGD
Loss	Binary cross entropy	Binary cross entropy	Binary cross entropy	Binary cross entropy	Binary cross entropy	Binary cross entropy
Epochs	500	500	500	500	500	1000
Flipping	True	True	True	True	True	True
Rotation range	40	40	40	40	40	40
Width/height shifting	0.1	0.1	0.1	0.1	0.1	0.1
Shear range	0.1	0.1	0.1	0.1	0.1	0.1
Zoom range	0.2	0.2	0.2	0.2	0.2	0.2

The article "Research on Classification of COVID-19 Chest X-Ray Image Modal Feature Fusion Based on Deep Learning" was published in 2021. Journal: J Healthc Eng.

**Table 3:** Summary of the pretrained convolutional neural network architecture used in this study.

Pretrained model		Input size	Layers	Size (MB)	Parameters (M)
ResNet50		224 × 224	50	98	23.52
ResNet152		224 × 224	152	232	60.42
Xception		299 × 299	126	88	22.91
InceptionResNetV2		299 × 299	572	215	55.87
Model 1	ResNet50	224 × 224	50	98	23.52
	Xception	299 × 299	126	88	22.91
	InceptionV3	224 × 224	159	92	23.85
Model 2	DesenNet201	224 × 224	201	80	20.24
	VGG19	224 × 224	19	549	143.67
	Xception	299 × 299	126	88	22.91
	ResNet152	224 × 224	152	232	60.42
	InceptionResNetV2	299 × 299	572	215	55.87

**Table 4:** Convolutional neural network architecture classification evaluation index score.

CNN	Index			
	Accuracy (%)	Precision (%)	Recall (%)	F1-score (%)
ResNet50	93.17	95.00	94.43	93.82
ResNet152	93.39	95.87	94.84	95.11
Xception	94.39	95.79	93.86	94.46
InceptionResNetV2	90.22	95.06	91.02	92.22
Model 1	94.76	95.45	96.02	94.99
Model 2	**96.00**	**96.10**	**96.42**	**95.50**

**Table 5:** Comparative computational time of convolutional neural network architectures.

Architectures	Training time (s)	Testing time (s)
ResNet50	418.91	58.87
ResNet152	472.65	61.05
Xception	440.46	61.60
InceptionResNetV2	560.20	52.44
Model1	725.99	61.48
Model2	1503.67	138.66

**Table 6:** Comparative study of the proposed model 2 with existing works with respect to accuracy, precision, recall and F1-score.

Author	Type of images	Architecture	Classes	Accuracy (%)	F1-score (%)	Precision (%)	Recall (%)
Sethy and Behera [20]	Chest X-ray	ResNet50 + SVM	2	95.33	95.34	—	—	
Hemdan et al. [31]	Chest X-ray	VGG19	2	90.00	90.00	91.50	90.00	
		DenseNet201	2	90.00	90.00	91.50	90.00	
Kumar et al. [17]	Chest X-ray	DeQueezeNet	2	94.52	—	90.48	96.15	
Jaiswal et al. [34]	Chest X-ray	COVIDPEN	2	**96.00**	94.00	92.00	96.00	
Ismael and Şengür [30]	Chest X-ray	ResNet50 + SVM	2	94.70	94.79	—	91.00	
Das [33]	Chest X-ray	DenseNet201 + Resnet50V2 + Inceptionv3	2	91.62	—	—	95.09	
Sahinbas and Catak [32]	Chest X-ray	VGG16	2	80.00	80.00	80.00	80.00	
This study	Chest X-ray	Model 2	2	**96.00**	**95.50**	**96.10**	**96.42**	

## Data Availability

The image experiment data used to support the study are available from the corresponding author upon request.
